# Additive Manufacturing Applications on Flexible Actuators for Active Orthoses and Medical Devices

**DOI:** 10.1155/2019/5659801

**Published:** 2019-03-24

**Authors:** Michele Gabrio Antonelli, Pierluigi Beomonte Zobel, Francesco Durante, Terenziano Raparelli

**Affiliations:** ^1^Department of Industrial and Information Engineering and Economics, University of L'Aquila, via G. Gronchi n. 18, 67100 L'Aquila, Italy; ^2^Department of Mechanical and Aerospace Engineering, Politecnico di Torino, Corso Duca degli Abruzzi 24, 10129 Torino, Italy

## Abstract

This paper describes the results of research projects developed at the University of L'Aquila by the research group of the authors in the field of biomedical engineering, which have seen an important use of additive manufacturing technologies in the prototyping step and, in some cases, also for the realization of preindustrialization prototypes. For these projects, commercial 3D printers and technologies such as fused deposition modelling (FDM) were used; the most commonly used polymers in these technologies are acrylonitrile butadiene styrene (ABS) and polylactic acid (PLA). The research projects concern the development of innovative actuators, such as pneumatic muscles and soft pneumatic actuators (SPAs), the development of active orthoses, such as a lower limb orthosis and, finally, the development of a variable-stiffness grasper to be used in natural orifice transluminal endoscopic surgery (NOTES). The main aspects of these research projects are described in the paper, highlighting the technologies used such as the finite element analysis and additive manufacturing.

## 1. Introduction

The authors have been engaged for several years in the development of innovative nontraditional actuators, and some of the research conducted on nontraditional pneumatic actuators, for example, for safety reasons, when the movements must take place avoiding that the moving parts constitute a danger to user, will be illustrated in this article. This is the case in the medical sector of assistive and rehabilitation devices, for example, an active orthosis, in which the patient interfaces directly with the device that has an autonomous movement capacity. In these cases, it is necessary that the actuator is intrinsically safe; therefore, it must not constitute a rigid system in movement but rather present adequate compliance for a greater system safety because this minimizes the risk of injury. Several researchers have developed compliant actuators able to perform a bending or a rotary movement and suitable for use in the biomedical and/or robotic field. These actuators are made of an elastomeric material and are pneumatically powered. Different solutions are proposed for deformation: an element of appropriate shape made only of soft material or the combination of an element in soft material with a reinforcement of adequate internal stiffness. In [1], two categories of soft pneumatic actuators (SPAs), the bending SPA and the rotary SPA, are presented and characterized and a procedure for the design of the types of actuators shown is described. In [2], the concept of assembling modular units of fabric-based rotary actuators for the construction of soft pneumatic structures, interesting for the realization of gripping systems with performances suitable for different types of objects, is illustrated. In the following sections, the term SPAs will be used for these nontraditional pneumatic actuators. The SPAs shown here are made of silicone rubber or natural lattice, due to their high deformability and simplicity of processing, inside which one or more chambers are obtained to contain the compressed air. When the latter is sent into the chamber, the structure deforms symmetrically or asymmetrically, if stiffness elements have been used (which can also be used to control the maximum deformation) or in the case of different thicknesses of the elastomeric material, as shown in Figure 1. The external load is applied through contact with the deformable surfaces. The power-to-weight ratio is higher than traditional actuators because they are very light materials. The force developed depends on the dimensions of the deformable chamber, the compressed air pressure value, the magnitude of the deformation caused, and the material used.

The intrinsic yielding of the elastomeric material makes these SPAs suitable for applications in the biomedical sector and makes it possible to realize actuators with geometries developed according to the specific application. These actuators require, for their realization, the preparation of a technological setup with the design and production of molds to which the silicone compound is poured, which allows the coupling of the half-shells. For the molds of various types of actuators realized, the additive manufacturing technology is frequently used. This technology has allowed the rapid and economic realization of the molds and the possibility of a simple optimization of the process even when it was necessary to modify the mold for a new realization. The properties of the polymeric materials used in 3D printers, such as ABS and PLA, meet the necessary strength and quality specifications, such as machining tolerances and surface finish, and they are easily operated with the usual design tools such as finite element analysis. Computer-aided design and finite element analysis have been among the most used tools for designing and sizing these innovative actuators and the manufacturing process. This paper shows some original development of SPAs, including applications in biomedical engineering, and of pneumatic muscle actuators, which are made up of elastomeric materials too. The McKibben pneumatic muscle is the most common type of braided muscle [3], and it will be discussed here. It is made of an inner elastomer tube surrounded by a braided shell and two ends. The straight fibres pneumatic muscle received less interest from the researchers [4], and it is formed by an elastomer tube inside in which there is an axial texture of cables, from one end to the other, and externally by circumferential rings that constrain the radial expansion. For both types of pneumatic muscles, the air inlet causes a radial expansion followed by an axial contraction of the heads, which allows an external traction work. This paper will also describe the research activity that led to the design and prototype realization of a remote-controlled surgical grasper, and of its variable-stiffness actuation (VSA) system, for whose technological development, the additive manufacturing was used. The robotics for the NOTES, also called natural orifice transluminal endoscopic robotic surgery (NOTERS), requires specific and customized solutions, such as a snail-like robot and the variable-stiffness actuation (VSA) implementation proposed in [5, 6]. Snail architecture uses a chain of elements connected to each other: the driver is placed near each joint, and the end effector can be guided with high dexterity in the peritoneal cavity. The VSA is recommended for developing high-performance devices for NOTERS, where intrinsic safety is required for both involuntary impact with internal organs and gripping, avoiding any potential damage to the soft tissue that is grasped. The use of SPA in the surgical gripper has proved to be very useful for the necessity of the VSA and for the extreme compactness required. With the NOTES, the abdominal cavity is reached in the absence of external incisions, exploiting the natural cavities such as the mouth, the rectum, and the vaginal conduit.

## 2. Materials and Methods

About the material used for soft pneumatic actuators and pneumatic muscles, since the constitutive law of the elastomeric material is nonlinear, as well as the behaviour of the air, being a compressible fluid, it is very complex to identify analytical correlations, assigned a geometry, among the deformation, the developed force and the pressure within the actuator chamber. Therefore, for the design of the actuators, the numerical modelling by the finite element method is carried out and, in some cases, for pneumatic muscles, the dimensional analysis is carried out, which allowed building a design graph based on three dimensionless parameters, which contain the quantities that influence the behaviour of the actuator. Several authors have developed models of pneumatic muscles of the braided type with the finite element method: the nonlinearity of the rubber tube has been simulated with the Mooney–Rivlin formulation with two coefficients as the mechanism for transferring the load to the braided shell [7]. Some authors [8] have proposed a nonlinear model to analyze the relationship between different muscles arranged in parallel and the total contraction ratio of each of them. This model examined geometric nonlinearity, while the behaviour of the rubber material was considered linear. Other authors [9] proposed a model to optimize the angle of the braided shell, and in [10], a method of quantitative optimization of the project is shown. The analysis of the scientific literature highlights the lack of a numerical model of the braided pneumatic muscle that is built on the real geometrical characteristics of the braided shell, as it is commercially available. In these models, the braided shell is analysed with average parameters available in the literature. The finite element model of the braided pneumatic muscle developed by the authors has been experimentally validated [11]. The model developed is nonlinear and based on real muscle parameters. It is proposed to predict the muscle behaviour and act as a reliable design tool. Several prototypes have been made of this muscle, and they have been applied in research projects for the development of orthoses. In Figures 2(a)–2(c), an example of numerical results of an isotonic test simulation, based on the model proposed, is shown. A research work was also carried out for straight fibres pneumatic muscles [12], and in Figure 2(d), an example of a characteristic graph obtained with the design curve is shown together with the curve required by the designer (traction force *F* vs. shortening Δ*L*) for a biomedical application.

The soft pneumatic actuators (SPAs), the straight fibres, and the braided pneumatic muscles require the experimental identification of the constitutive law of the elastomeric material used (e.g., Silastic *E* of Dow Corning). In the presence of actuator symmetries, the geometry modelled by the finite elements can represent half or a quarter of the entire geometry (Figure 3).

Usually, it is sufficient to create two models: a model that simulates the isometric test conditions and the one that simulates isotonic ones. In the first case, with constant deformation, the force value developed by the actuator is correlated to the air pressure; in the second, at constant load, the deformation of the actuator correlates with the air pressure. The finite elements used for the silicone rubber modelling are of the brick type, and the elastomeric material is modelled by the Mooney–Rivlin formulation with two coefficients. Once the actuator has been sized, the first step is the designing of the mold, made of polymeric materials by additive manufacturing. Then, the preparation of the silicone rubber starts as follows: before the catalysis takes place, the rubber has a very fluid consistency and is easily pourable. Before casting, it is advisable to proceed with the removal of air bubbles present in the silicone rubber mix, to avoid inclusions inside the actuator. Thus, the casting is carried out. Depending on the type of SPA, the construction can take place in a single casting or in successive phases. The second mode occurs when a metal plate or a bar is incorporated into the actuator to limit deformation in an assigned direction or when multichamber actuators are to be made. Thus, the construction of a first layer of the actuator is carried out. And the mixture is expected to start to solidify, and the high stiffness material is deposited; then, a second casting is carried out; the second casting is expected to start to solidify and the material for the construction of the chamber is laid below another casting until the entire mold is filled. Typically, the construction of the chamber is carried out by a sheet of paper or by wax, according to requirements. An example of embodiment of a square-shaped SPA is shown in Figure 4. The conduit for air supply and discharge can be integrated with the actuator (in this case, it is made of silicone rubber during the casting process) or the mold is designed with a cavity inside the actuator, where the valve will be placed.

## 3. Results and Discussion

### 3.1. Actuators and Active Orthoses

The types of pneumatic actuators presented here belong to two different families: pneumatic muscles and soft pneumatic actuators (SPAs). The former have been the subject of research activities and find space in some industrial applications, as they are available in the automation components market; the latter are not present in the market but are often designed ad hoc and integrated into commonly used devices such as blood pressure measurement systems and other medical devices, such as car seats and massage chairs. Two types of pneumatic muscles have been developed [11, 12]: straight fibres and braided, also known as McKibben muscle. The straight fibres pneumatic muscle (Figure 5(a)) is made of a silicone cylindrical chamber in the wall in which a cage consists of 40 Kevlar threads, arranged longitudinally and held in position by two end rings, in which one is buried inside the silicone and the other is connected to the head that contains the air supply/discharge pipe. The pneumatic and mechanical seal is ensured by means of clamping systems with the tube at the heads. To limit the radial deformation of the muscle, metal circumferential rings are arranged externally of the cylindrical chamber. The pneumatic muscle of the McKibben type (Figure 5(b)) is formed by using a cylindrical chamber made of the elastomeric material, a sheath consisting of a rhomboidal mesh that covers the chamber externally, and two heads which have the function of isolating the chamber, blocking the sheath on the outside of the chamber, and allowing the anchorage of the muscle to the device. On one of the two heads, the air supply/discharge hole is made. The sheath is of the braided type and has a cylindrical shape: the wires, in polyamide, are placed side by side in numbers of six and wound to form 42 spirals that create rhomboidal meshes. Sending air into the chamber causes an increase in volume so that the outer surface of it comes into contact with the outer sheath; the muscle contracts due to the high axial rigidity of the wires forming the sheath.  Table 1 shows the characteristics of the silicone muscles made. Pneumatic muscles have been used in research applications in the biomedical sector: those with straight fibres for the movement of an anthropomorphic rehabilitation robot of the upper limb and with the braided muscles for the movement of an inferior and upper limb orthosis.

The active orthosis for inferior limb is a research project born with the aim of developing a solution to allow the elderly, and people with weak strength in the legs, to have a wearable device under the pants that can give them additional strength in the legs to allow them to get up from a sitting position. The result of this research activity [13] is an optimized prototype of a one degree-of-freedom lower limb orthosis with a light structure; it is made of carbon fibre and naturally activated with a sensor that detects the contraction of the quadriceps femoris of the user.

This type of command allows the orthosis to be activated even when the user is sitting, avoiding the impact on the seat that can cause traumas. The carbon fibre structure is made in laboratories using a fibre sock, suitable for making tubular structures with a diameter from 20 to 45 mm, impregnated with epoxy resin through an ABS mold manufactured by additive manufacturing. The mold is hollow and made of two shells. To allow the correct polymerization of the fibre inside the mold in the desired thicknesses, a rubber cylinder was inserted and subsequently filled with pressurized air so as to obtain an adequate thrust of the fibre against the inner surface of the mold. During the polymerization, the vertical arrangement was used which guaranteed the best surface finish of the product. In Figure 6(a), one of the orthotics molds, 244 mm long, is visible, while in Figure 6(b), the resin application on the socks of carbon fibre, after having inserted them into the rubber cylinder, is shown.

Figure 7(a) shows the rubber cylinder coated by the socks into the mold, while in Figure 7(b), the manufactured tube in carbon fibre is shown and, finally, the prototype of orthosis assembled is shown in Figure 8. The sock in carbon fibre has a thickness of about 0.5 mm and, to obtain a thickness of about 2 mm for the structure, it was necessary to use 4 layers of sock, at whose ends an adhesive was applied to keep the fibres in the desired arrangement. The impregnation with the epoxy resin takes place after the insertion of the first sock on the rubber cylinder and continued after the insertion of each of the following carbon fibre socks. On the inside wall of the mold, it was necessary to apply a detaching wax to prevent adhesion between the carbon fibre and the ABS mold. After the mold has been closed, the cylinder has been brought to a pressure of 1 bar and therefore kept in the oven for a thermal cycle of 20 hours at 45°C. Once the polymerization was finished and the product was extracted, an acrylic finishing layer was applied.

Square-shaped SPAs were made and inside which a chamber is located to fill compressed air. The planar geometry of the SPAs can be different depending on the application: square, rectangular, circular, semicircular, and toroidal. The geometry of the chamber reproduces the geometry of the external shape of the actuator, but in some cases, it may be different. Regardless of the profile of the perimeter, the actuators are characterized by having the nondeformable perimeter. Inside the SPA can be located a single volume or several volumes, each with its own air supply/discharge channel or connected to each other but with a single air channel. Simple types of single-chamber SPA have been designed for applications in the medical field. A series of actuators has been installed inside a scoliosis brace in order to apply a push action on the spine [14]. These are SPAs with a single square-shaped chamber. The chamber deforms unilaterally, having placed a metal plate at the other end. The air supply/exhaust channel was obtained by means of a common tire tube valve for bicycle use and mounted on the side where the metal plate is present, as shown in Figure 9.

The therapist using a manual bag to inflate adjusts the air pressure for each soft pneumatic actuator. A SPA with several chambers, each having its air supply/discharge channel, has been designed and manufactured for the massage device shown in Figure 10 [15].

The multichamber SPA, mounted on a structure that is worn by the subject and which is in contact with the lumbar segment of the spine, applies a compression action. The intensity of this thrust is adjusted by varying the pressure value inside the chamber. Each multichamber SPA has 6 small actuators. The actuator is deformed from one side; on the opposite side, a metal plate is placed and the silicone air supply/discharge channel is obtained. The massage device consists of 8 SPAs with a total of 48 actuators. By suitably filling the different volumes, the common massage techniques used by the physiotherapist are reproduced. The order of feeding the chambers and the pressure and the frequency of air supply/discharge are managed by a programmable logical controller. In Figure 11, the result of the characterization tests carried out on the multichamber SPA is shown. Similar technology has been used for developing an articulated finger for a gripper device [16] and for an active brace for the unloading of the lumbar spine [17]. The brace is made with two rigid elements, one lower and one upper, respectively, in contact with the iliac crests and with the thoracic sockets. Distancing the two elements from each other produces an unloading of the lumbar spine section. The movement of the rigid elements is entrusted to the actuators, interposed between them, and positioned at the sides of the user.

The SPAs with several chambers, located on different planes in a parallel disposition, joined together by a single air supply/discharge channel, and made of silicone rubber during the casting phase of the actuator, are shown in Figure 12(a). In Figure 12(b), the prototype of the active brace is shown, and the characteristic curve of strength *F* vs. displacement Δ*h* is shown in Figure 13.

Each multichamber SPA consists of 5 chambers of semicircular geometry, symmetrically deformable. The therapist using a manual bag to inflate adjusts the air pressure value, following the medical prescription.  Table 2 shows the dimensional and functional characteristics of the realized silicone rubber SPAs.

### 3.2. Medical Devices

Additive manufacturing is spreading more and more for manufacturing medical devices with the aim of using them as customized prostheses that the single surgeon adapts and prints for the specific patient. At present, the critical issues are related not so much to static loads as to cyclic loads, as was shown for load-bearing implants [18]. By using the additive manufacturing for the soft pneumatic actuator (SPA), the research project on a surgical grasper has been carried out. It has the focus in the natural orifice transluminal endoscopic surgery (NOTES) where the abdominal cavity is reached, exploiting the natural cavities such as the mouth, the rectum, and the vaginal conduit. The advantage of this type of surgery is represented by the absence of scars, the reduction of the recovery time, and the recovery of the patient. Due to the limitations of current surgical instruments for laparoscopy, NOTES must necessarily resort to robotic systems operated by the surgeon and become natural orifice transluminal endoscopic robotic surgery (NOTERS). In the NOTERS, collision safety can be ensured by yielding devices that reduce the effects of the impact on the patient; performance depends heavily on the interaction of the operating mechanics of the surgical instrument with the control system. To meet both requirements, several solutions have been proposed: decoupling the inertia of the instrument implementation system from the inertia of its structure, by means of an elastic transmission; the use of a pair of actuators, one of which is used in low-frequency and the other in high-frequency applications; the use of variable-stiffness systems [19], which is the solution chosen for the developed prototype of the surgical grasper presented here with the focus on the SPA. The main technical specifications underlying the implementation of this surgical grasper, for the type of grip adopted, are as follows: variable stiffness, ability to exert a maximum force equal to 11.50 N, and ability to allow a maximum displacement of the rod of the subassembly of 2.4 mm. Furthermore, the outer diameter of the entire prototype implementation subassembly must not exceed 12 mm. The operating principle of the SPA is shown in Figure 14(b). The solution developed for the implementation of a variable-stiffness device for the miniaturized graspers (Figure 14(a)) is pneumatic actuation by means of a SPA, made of silicone rubber, mounted in line, and arranged in agonist-antagonist position, as shown in Figure 15(b). The prototype of the gasper is shown in Figure 15(a).

These circular-shaped SPAs are characterized by having inside them an air chamber formed between two circular silicone rubber surfaces, connected to each other along the circumference: sending air into the chamber causes a deformation of the actuator, due to the silicone's compliance, which can occur at both the surfaces or only one, depending on the construction mode. The agonist-antagonist mode of the actuator system is necessary for opening and closing of the grasper. by acting on the air pressure inside the chambers, it is possible to control the stiffness of the transmission, as shown in Figure 14(b). The realization of the SPAs has been facilitated by the use of FDM technology of additive manufacturing with different materials, and the best results for the application have been obtained with the ABS. The designing of the actuators was carried out by means of numerical modelling by finite elements technique, also thanks to the know-how of the authors on the modelling of silicone rubber SPAs. Isometric models were simulated to derive the force developed by the actuator as a function of the pressure, for an assigned deformation. The optimal solution was provided by the actuator model characterized by an external diameter of 10 mm, a diameter of the deformable surface equal to 8 mm, and a thickness of the deformable surface equal to 1 mm. From the analysis of the results, it is observed that, for a typical stroke of 1.8 mm, only one actuator is able to exert a force equal to 7 N at 0.3 MPa, sufficient to close the clamp when the load is applied to it externally with a maximum load of 3 N. For the maximum stroke of 2.4 mm, the 0.3 MPa actuator exerts a force of 6 N. In compliance with the specifications, it was established to adopt a pair of SPAs for closing the clamp and a single SPA for opening. The latter requires a minimum of negligible force. The prototype grasper shown in Figure 15(a) was submitted to a campaign of laboratory validation tests that gave very positive results.

## 4. Conclusion

This paper shows the main results of the research activities carried out by the authors in the field of pneumatic muscles and soft pneumatic actuators for use in active orthoses and medical devices. In this field, a wide use was made of additive manufacturing technology, for the realization of the molds, and of computer-aided design tools and of the finite element method for designing and sizing of the actuators and devices in which they have been applied. The actuators presented are pneumatic muscles and square-sized and circular-sized SPAs. The latter were applied to a scoliosis brace, to a massage device, to a spinal unloading brace, and to a surgical grasper, the main results of which have been described in the paper. The application of additive manufacturing in the construction of molds for the manufacturing of the prototype of lower limb orthosis in carbon fibre is also presented. The results obtained are of scientific interest, and the applications presented demonstrate the effectiveness of additive manufacturing technology in the field of assistive devices and rehabilitation systems, as well as computer-aided design and the finite element method. The research work is in progress for some applications with the study of other elastomers such as natural latex, which allow a better resistance to fatigue than silicone.

## Figures and Tables

**Figure 1:** Mode of SPA deformation: (a) symmetrical; (b) unilateral, by inserting stiffness material or (c) through increase in thickness.

**Figure 2:** Numerical results of an isotonic test simulation with the braided pneumatic muscle model: (a) rest muscle; (b) during shortening; (c) at maximum inflation speed (side view). Graph obtained by connecting the design curve of the straight fibre pneumatic muscle together with the curve desired by the designer (d).

**Figure 3:** Example of a SPA prototype with an output of the finite element model.

**Figure 4:** Steps of manufacturing a square-shaped SPA: after solidification of the first silicone layer, (a) deposition of an element with high rigidity; (b) deposition of a second layer of silicone; (c) deposition of a sheet of paper or wax for the realization of the volume; (d) filling the mold with another layer of silicone.

**Figure 5:** Prototypes of pneumatic muscles developed: straight fibres (a) and braided (b), also known as McKibben muscle.

**Figure 6:** Mold shells made of ABS by additive manufacturing (a) and an impregnation step of the carbon fibre braided with the resin (b).

**Figure 7:** Mold of the pneumatic core coated with the impregnated carbon fibre socks (a) and the result obtained after polymerization (b).

**Figure 8:** Prototype of lower limb orthosis made of carbon fibre with aluminum joints.

**Figure 9:** Square-shaped SPA (a) and application in a brace for scoliosis with the thrusts in specific points of the spine (b).

**Figure 10:** Spine massage device (a) and details of the multichamber SPA and of the processing mold (b).

**Figure 11:** Results of characterization tests on multichamber SPA: isotonic displacement vs. pressure and isometric force vs. displacement.

**Figure 12:** Multichamber SPA (a) and the prototype of the active brace (b).

**Figure 13:** Characteristic curve of the brace built in the laboratory as strength *F* vs. displacement Δ*h* at different pressure values.

**Figure 14:** Axonometric view of the developed surgical grasper (a) and the principle of operation of the actuation module (b).

**Figure 15:** Prototype of NOTERS grasper realized (a) and view of the circular-shaped SPA (b).

**Table 1:** Main characteristics of silicone pneumatic muscles made.

Type of pneumatic muscle	Length (mm)		External diameter (mm)		*P*_max_ (bar)	*F*_max_ (N)
	At rest	At maximum contraction	At rest	At maximum contraction		
Straight fibres	300	217	30	91	1.5	1000
Braided	285	209	30	54	2.5	500

**Table 2:** Main features of the silicone rubber SPAs.

Field of application	Dimensions, *b* × *h* × *s* (mm^3^)	Type of deformation	Maximum deformation (mm)	*P*_max_ (bar)	*F*_max_ (N)
Brace for scoliosis	80 × 80 × 10	Monolateral	40	0.6	100
Grasper	60 × 40 × 10	Symmetrical	14	0.8	90
Massage device	44 × 36 × 9^*∗*^ 104 × 123 × 9^*∗∗*^	Monolateral	10	1	30
Brace for unloading the spine	128 × 88 × 6^*∗∗∗*^	Symmetrical	20	0.5	800

^*∗*^Dimension of the single-channel SPA; ^*∗∗*^dimension of the multichannel SPA; ^*∗∗∗*^external radius × internal radius × thickness.

## Data Availability

The authors state that the results cited in this research work are related to numerical simulations and to experimental test campaigns. Data supporting the findings of this study are available from the corresponding author [PBZ] on request.
